The article "Meta-Analysis of Low Density Lipoprotein Receptor (LDLR) rs2228671 Polymorphism and Coronary Heart Disease" was published in 2014. Journal: Biomed Res Int.

# Meta-Analysis of Low Density Lipoprotein Receptor (*LDLR*) rs2228671 Polymorphism and Coronary Heart Disease

**DOI:** 10.1155/2014/564940

**Published:** 2014-05-12

**Authors:** Huadan Ye, Qianlei Zhao, Yi Huang, Lingyan Wang, Haibo Liu, Chunming Wang, Dongjun Dai, Leiting Xu, Meng Ye, Shiwei Duan

**Affiliations:** ^1^Zhejiang Provincial Key Laboratory of Pathophysiology, School of Medicine, Ningbo University, Ningbo, Zhejiang 315211, China; ^2^The Affiliated Hospital, School of Medicine, Ningbo University, Ningbo, Zhejiang 315211, China; ^3^Yinzhou People's Hospital, School of Medicine, Ningbo University, Ningbo, Zhejiang 315040, China; ^4^Bank of Blood Products, Ningbo No. 2 Hospital, Ningbo, Zhejiang 315010, China

## Abstract

Low density lipoprotein receptor (LDLR) can regulate cholesterol metabolism by removing the excess low density lipoprotein cholesterol (LDL-C) in blood. Since cholesterol metabolism is often disrupted in coronary heart disease (CHD), *LDLR* as a candidate gene of CHD has been intensively studied. The goal of our study is to evaluate the overall contribution of *LDLR* rs2228671 polymorphism to the risk of CHD by combining the genotyping data from multiple case-control studies. Our meta-analysis is involved with 8 case-control studies among 7588 cases and 9711 controls to test the association between *LDLR* rs2228671 polymorphism and CHD. In addition, we performed a case-control study of *LDLR* rs2228671 polymorphism with the risk of CHD in Chinese population. Our meta-analysis showed that rs2228671-T allele was significantly associated with a reduced risk of CHD (*P* = 0.0005, odds ratio (OR) = 0.83, and 95% confidence interval (95% CI) = 0.75–0.92). However, rs2228671-T allele frequency was rare (1%) and was not associated with CHD in Han Chinese (*P* = 0.49), suggesting an ethnic difference of *LDLR* rs2228671 polymorphism. Meta-analysis has established rs2228671 as a protective factor of CHD in Europeans. The lack of association in Chinese reflects an ethnic difference of this genetic variant between Chinese and European populations.

## 1. Introduction

Coronary heart disease (CHD) is a complex disease caused by an insufficient blood flow inside the coronary vessels [1]. The blockage of the arteries is often caused by the plaque accumulated in the wall of arteries. The plaque is formed by excess low density lipoprotein cholesterol (LDL-C) in blood that dramatically increases the risk of CHD [2]. Low density lipoprotein receptor (LDLR) plays a key role in the regulation of cholesterol metabolism by removing excess LDL-C in blood [3, 4].

CHD is caused by both environmental and genetic factors [5]. Variations of genes involved in lipoprotein and lipid metabolism are playing an important role in the susceptibility of CHD [6].* LDLR* gene mutations can lead to deficiency or abnormality of LDLR in the cell membrane surface and thus disrupt lipid metabolism [4].* LDLR* gene mutations are known to cause familial hypercholesterolemia (FH) [2] that is an important risk factor of CHD and other atherosclerotic diseases [7]. Recent genome-wide association studies (GWASs) showed that* LDLR* gene mutations were significantly associated with the abnormal blood lipid levels and CHD [8, 9]. Among the* LDLR *polymorphisms, rs2228671 was associated with LDL-C levels and CHD in German and British populations [10–14]. However, discrepancies were also shown in the association of* LDLR *rs2228671 with CHD in Italians and Germans [15, 16].

The article "Meta-Analysis of Low Density Lipoprotein Receptor (LDLR) rs2228671 Polymorphism and Coronary Heart Disease" was published in 2014. Journal: Biomed Res Int.

Meta-analysis is able to combine and review the results from previous studies [17, 18]. Meta-analysis improves the power of comprehensive statistics by pooling the data from different studies. In the present study, we performed a meta-analysis of* LDLR *rs2228671 polymorphism with CHD among 17299 individuals in 8 studies.

## 2. Material and Methods

### 2.1. Retrieval of Studies and Selection Criteria

We systematically search available studies from 2003 to 2013 in PubMed (English), CNKI, and Wanfang (Chinese). Keywords were “coronary heart disease” or “coronary artery disease” or “myocardial infarction” combined with “*LDLR*” or “low density lipoprotein receptor” or “rs2228671” and “polymorphism” or “genetic association.” The inclusion criteria for the studies involved in this meta-analysis met the following criteria: (1) case-control study about* LDLR* rs2228671 polymorphism; (2) case-control study with genotyping or allelic information, or odd ratio (OR) with 95% confidential interval (CI).

### 2.2. Data Extraction

Data included in this meta-analysis was extracted independently from all studies using the same standard protocol by two reviewers (HY and YH). The inclusion criteria of our meta-analysis were as follows: first author's name, publication year, ethnicity, numbers of cases and controls, genotype distribution, and OR with 95% CI.

### 2.3. Patients and Controls

The study protocol was approved by the ethical committee of School of Medicine, Ningbo University. A total of 162 cases and 113 controls were recruited in this study from the Affiliated Hospital of Ningbo University. All the participants in this study have signed the informed consent forms. All the 275 individuals underwent coronary angiography and were categorized into CHD patients and non-CHD controls according to our previous descriptions [5, 19]. All the participants enrolled in this study were Han Chinese residing in or near Ningbo city. None of individuals in this study had congenital heart disease, cardiomyopathy and severe liver, or kidney disease.

The article "Meta-Analysis of Low Density Lipoprotein Receptor (LDLR) rs2228671 Polymorphism and Coronary Heart Disease" was published in 2014. Journal: Biomed Res Int.

### 2.4. SNP Genotyping

Genomic DNA was isolated from peripheral blood lymphocytes using standard phenol-chloroform method and then was stored in TE buffer. All DNA samples were amplified by polymerase chain reaction (PCR). PCR was denatured at 94°C for 15 s, followed by 45 cycles of denaturation at 94°C for 20 s, annealing for 30 s at 56°C, extension at 72°C for 1 min, and a final extension at 72°C for 3 min. DNA amplification and genotyping was performed on the SEQUENOM Mass-ARRAY iPLEX platform according to the manufacturer's instructions [5].

### 2.5. Statistical Analyses

Hardy-Weinberg equilibrium (HWE) was examined by the Arlequin program (version 3.5) [20]. The differences in the genotype and allele frequencies between cases and controls were analyzed by the CLUMP22 software with 10,000 Monte Carlo simulations [21]. Power analysis was performed by Power and Sample Size Calculation software [22]. Meta-analysis was made by REVMAN 5.0 (Cochrane Collaboration, Oxford, United Kingdom) and Strata 11.0 software (Strata Corporation, College Station, TX) [23, 24]. Publication bias was evaluated by Begg and Egger regression tests [25]. The combined ORs with 95% CI values were calculated by either fixed-effect or random-effect method [26]. A two-tailed *P* value of 0.05 or lower was defined to be statistically significant.

## 3. Results

We systematically searched in PubMed, CNKI, and Wanfang from 2003 to 2013, and selected a total of 57 literatures after removing the duplicated publications (Figure 1). According to the descriptions in the titles and abstracts, we excluded 26 irrelevant literatures, 6 literatures on other variants, and 12 literatures on other diseases. In addition, 1 literature without sufficient case-control genotyping data and 5 literatures without detailed SNP information were also removed. At last, 6 literatures [11–16] on 7 case-control studies were harvested in our meta-analysis (Table 1). Furthermore, we performed a case-control study in Han Chinese population, and it was later included in our meta-analysis.

Genotype distribution of rs2228671 in our case-control study met HWE for both CHD cases and non-CHD controls (*P* > 0.05), indicating that our case-control study had a well-characterized random sampling. Our case-control study suggested that* LDLR* rs2228671-T allele was rare in Chinese population (cases: 2%; controls: 1%), and this agrees with the frequency in HapMap Chinese Han in Beijing (CHB) population (0–2%). No significant difference in the genotype distribution between CHD cases and non-CHD controls are revealed in all samples (*P* > 0.05; Table 2) and in the subgroup analysis by gender (*P* > 0.05; Table 2). In summary, our case-control study showed that there was no association between* LDLR* rs2228671 and CHD in Chinese. However, significant association was found between* LDLR* rs2228671 and CHD in European population (*χ* ^2^ = 20.59, *P* < 0.0001 by genotype; *χ* ^2^ = 20.26; OR = 1.180, 95% CI = 1.098–1.269, *P* < 0.0001 by allele; Table 3). Using the fixed-effect method, our meta-analysis contained 7,588 CHD patients and 9,711 controls from German, British, Italian, and Chinese populations. As shown in Figure 2, significant association was observed between rs2228671 and CHD (*P* = 0.0005, OR = 0.83, and 95% CI = 0.75–0.92). In addition, no heterogeneity among the studies was included in this meta-analysis (*I* ^2^ = 0%; Figure 2). Furthermore, no obvious visual evidence of publication bias in the meta-analysis was shown by funnel plot (*P* > 0.05; Figure 3).

The article "Meta-Analysis of Low Density Lipoprotein Receptor (LDLR) rs2228671 Polymorphism and Coronary Heart Disease" was published in 2014. Journal: Biomed Res Int.

## 4. Discussion

Aberrant LDLR level in blood can cause abnormal cholesterol metabolism [2]. As the main pathogenic gene of FH,* LDLR* gene is associated with multiple vascular diseases [15, 16, 27]. Polymorphisms of* LDLR* gene were associated with type 2 diabetes [28] and hypertension [29] that also related to CHD. Recently, a handful of* LDLR* polymorphisms have been studied in CHD, including those (rs14158, rs3826810, rs1433099, rs2738464, rs2738465, and rs2738466) in the 3′-untranslated region (3′-UTR) and rs2228671 in second exon [30–32]. SNPs in first intron (rs6511720) and 5′ flanking region (rs17248720) of* LDLR* gene were closely related to both LDL-C and CHD [33, 34]. Rs1433099 and rs2738466 in the 3′-UTR of* LDLR* were reported to be associated with baseline lipids in American population [32]. The T allele of rs2228671 polymorphism was associated with higher FVIII:c levels. In addition, LDLR rs2228671 may be regulated FVIII:c levels and associated with the independence risk factor (plasma lipids) of CHD [16].

Our meta-analysis among 17299 individuals showed that rs2228671-T allele reduced the risk of coronary heart disease in the combined samples from German, British, Italian, and Chinese populations (OR = 0.83, *P* = 0.0005). Furthermore, rs2228671-T allele frequencies in the meta-analysis among German, British, and Italian populations were 7–12.2% that is similar to 10% in HapMap CEU population. However, rs2228671-T allele frequency is 0% in HapMap CHB population and 0.9% in the controls of our study. Due to the rare allele of* LDLR* rs2228671 in our samples, the power of our case-control study was only 5.1%, in contrast of 100% in the present meta-analysis. This suggests that a lack of association in our case-control study may largely be explained by the insufficient power for this rare polymorphism and the small sample size. Future investigation on other common* LDLR *polymorphisms is worth being performed in a large Chinese cohort.

The article "Meta-Analysis of Low Density Lipoprotein Receptor (LDLR) rs2228671 Polymorphism and Coronary Heart Disease" was published in 2014. Journal: Biomed Res Int.

Human* LDLR* is about 43 kb in length and has 1367 active polymorphism. As shown in our study, the allele frequency of rs1122608-T is much lower than those in the European studies; suggesting a cross-population comparison of this polymorphism may help one understand the role of* LDLR* in different ethnic population. Meanwhile, the previous tested* LDLR* rs1122608 polymorphism did not yield a significant result (*P* = 0.148) [35], in contrast to a significant result of rs2228671 in the current study (*P* = 0.0005). This suggests rs2228671 and rs1122608 might exert different contributions to the risk of CHD.

There were several limitations in our study as follows. Firstly, most of the involved individuals in our meta-analysis were Europeans; thus our result might not be applied to other populations such as Chinese. Secondly, although we had no evidence of the publication bias in our meta-analysis, we cannot exclude the possibility of existing potential bias upon reporting the studies without significant association results. Last but not least, the power of our case-control study in Chinese is only 5.1%. The negative result of rs2228671 might not represent for other variants of* LDLR *gene in Chinese population.

In conclusion, the meta-analysis demonstrated that the* LDLR* rs2228671-T allele is a protective factor of CHD in Europeans. However, the case-control study showed no significant association of* LDLR* rs2228671 with CHD in Han Chinese population.

## Figures and Tables

**Figure 1:** Flowing chart of selection publications in the current meta-analysis.

**Figure 2:** Meta-analysis of rs2228671 with CHD.

**Figure 3:** Publication bias analysis of 8 studies in the meta-analysis. The Begg's funnel plot and the Egger's publication bias plot test also indicated little evidence of publication bias among studies of rs2228671 and CHD risk (Begg, *P* = 0.536; Egger, *P* = 0.515).

**Table 1:** Characteristics of the association studies between rs2228671 and CHD.

Author and year	Ethnic group	Genotype (CC/CT/TT)		*P*-allele
		Cases	Controls	
Ortlepp et al. (2003) [11]	German	937/216/10	972/255/22	0.0453
Krawczak et al. (2006) [12]	German	1755/379/19	1840/474/25	0.0184
Samani et al. (2007) [13]	German	781/93/1	1417/224/3	0.0281
Samani et al. (2007) [13]	British	1578/322/13	2332/569/34	0.0051
Schunkert et al. (2008) [14]	German	236/43/2	224/61/5	0.0343
Erdmann et al. (2009) [15]	German	282/64/3	671/164/15	0.3333
Martinelli et al. (2010) [16]	Italian	549/134/9	227/61/3	0.73
Our study (2013)	Chinese	157/4/1	111/2/0	0.485

The article "Meta-Analysis of Low Density Lipoprotein Receptor (LDLR) rs2228671 Polymorphism and Coronary Heart Disease" was published in 2014. Journal: Biomed Res Int.

**Table 2:** Genotype and allele frequency distributionof* LDLR* gene rs2228671 polymorphism in cases and controls*.

Gender	Group	CC/CT/TT	*χ* ^2^	*P* (df = 2)	C/T	*χ* ^2^	*P* (df = 1)	OR (95% CI)
All	Cases	157/4/1	0.86	1	318/6	0.87	0.49	0.47 (0.09–2.36)
	Controls	111/2/0			224/2			

Male	Cases	113/2/1	0.51	0.77	228/4	NA	NA	0.49 (0.05–4.41)
	Controls	58/1/0			117/1			

Female	Cases	44/2/0	0.53	0.76	90/2	NA	NA	0.42 (0.04–4.71)
	Controls	53/1/0			107/1			

*NA represents not analyzed; rs2228671 meets HWE in all groups (*P* > 0.05).

**Table 3:** Genotype and allele frequency distributionof* LDLR* gene rs2228671 polymorphism in European population.

Gender	Group	CC/CT/TT	*χ* ^2^	*P* (df = 2)	C/T	*χ* ^2^	*P* (df = 1)	OR (95% CI)
European population	Cases	6218/1251/57	20.59	<.0001	13687/1365	20.26	<.0001	1.180 (1.098–1.269)
	Controls	7685/1808/107			17178/2022			
